# Pattern of condom use among clients at a Nigerian HIV Counseling and Testing Centre

**DOI:** 10.1186/1756-0500-6-289

**Published:** 2013-07-24

**Authors:** Samuel A Olowookere, Najeemdeen A Adeleke, Akinola A Fatiregun, Emmanuel A Abioye-Kuteyi

**Affiliations:** 1 Department of Community Health, Faculty of Clinical Sciences, College of Health Sciences, Obafemi Awolowo University, Ile-Ife, Nigeria; 2 Department of Obstetric and Gynaecology, Osun State University, Osogbo, Osun State, Nigeria; 3 Department of Epidemiology and Medical Statistics, Faculty of Public Health, College of Medicine, University of Ibadan, Ibadan, Oyo State, Nigeria

**Keywords:** Sexual behaviour, Condom use, HCT Centre, HIV/AIDS

## Abstract

**Background:**

Studies in Nigeria have shown that the main route of HIV transmission is sexual intercourse and that effective condom use protects people against infection. The objective of this study was to determine the pattern of condom use among clients of a friendly HIV Counseling and Testing (HCT) Centre in Osogbo southwestern Nigeria.

**Methods:**

This was a review of the HCT Centre records from 2006 to 2010 retrieving socio-demographic information, sexual behaviour, condom use and result of HIV testing. Data obtained were analyzed using descriptive and inferential statistics.

**Results:**

One thousand nine hundred and twenty-one client records were reviewed. The mean age of the study population was 35.4 (SD 10.5) years. The majority (53%) of the respondents were females, 232 (12%) were HIV positive, and 38.2% had multiple sexual partners. Only heterosexual vaginal sex was reported among the clients. Overall 45.2% of the clients did not use a condom in their last sexual act. Factors identified to be significantly associated with non-use of condoms were; younger age, having had higher education and positive HIV status.

**Conclusion:**

Unprotected heterosexual intercourse was common among the study population, indicating a need to step up HIV preventive programme through behavioural change communication strategy.

## Findings

## Background

The prevalence of Human Immunodeficiency Virus (HIV) in sub-Saharan Africa is the highest in the world [1]. As at the end of 2009, about 33.3 million people were estimated to be infected with HIV globally. Of these 22.5 million lived in sub-Saharan Africa with about 2.98 million in Nigeria [2]. Thus Nigeria ranked second to South Africa in terms of population of people living with HIV/AIDS in Africa [3]. Since the first case of AIDS in Nigeria was reported in 1986, the HIV/AIDS epidemic has continued to evolve with the antenatal clinic attendees sentinel surveillance surveys showing HIV prevalence rates of 1.8% in 1991; 5.8% in 2001; 4.4% in 2005; 4.6% in 2008 and 4.1% in 2010. Presently an estimated total of 3.1 million live with HIV/AIDS in Nigeria [2-4].

The leading route of HIV transmission in Nigeria is by heterosexual intercourse, accounting for 80% of the infections. The remaining 20% of infections occur mainly through mother-to-child and transfusion of infected blood and blood products [4]. Other modes of HIV transmission that are becoming important in Nigeria include men having sex with men, injecting and other drug users [5,6]. The drivers of the HIV epidemic in Nigeria included low risk perception, multiple concurrent partners, informal transactional and inter-generational sex, lack of effective services for sexually transmitted infections (STIs) and poor quality of health services. Gender inequalities, poverty and HIV/AIDS stigma and discrimination also significantly contributed to the continuing spread of the infection [6]. There are both increase and decrease in the HIV prevalence in Osun State over a time period between 2001 and 2010, 4.3% in 2001 to 1.2% in 2003, then 2% in 2005, 1.2% in 2008 and 2.7% in 2010 [7].

Evidence had shown that consistent correct use of condom has been widely recommended as a public health strategy worldwide against sexually transmitted infections, including heterosexual transmission of HIV infection [4,8,9]. The male latex condom is the single, most efficient, available technology to reduce the sexual transmission of HIV and other sexually transmitted infections. The use of condoms is recommended for individuals who have multiple partners, who have a primary partner who is infected, or whose partner’s serostatus is unknown [10]. However, no study has looked at the pattern of condom use among this sexually active population, highlighted the need for this study.

The objective of this study was to determine the pattern of condom use among clients of the Friendly HIV Counseling and Testing (HCT) Centre in Osogbo, southwestern Nigeria.

## Methods

The HCT Centre was established by the Osun State Government, Nigeria with the support of the United Nations Population Fund (UNFPA) in August 2005 to offer free HIV counseling and testing services including free condom distribution to people living in Osun State and beyond.

The Centre opens from 8:00 am to 4:00 pm Monday through Friday. It conducts free HIV counseling and testing services to the general public during important programmes such as the World AIDS Day and the annual Osun Osogbo Festival. It also provides free HIV counseling and testing to clients who visit the HCT Centre. Clients are attended to by nurse counsellors who carried out pre-test counseling after which the clients who consented have HIV screening and then post-test counseling which included discussing their test results. The information collected is entered into the client’s record form. HIV positive cases are referred to the nearby antiretroviral clinics situated at Ladoke Akintola University (LAUTECH) Teaching Hospital or State Hospital both located in Osogbo, whereas HIV negative clients are requested to come back in three months or anytime they become ill for a repeat HIV counseling and testing and are counseled on minimizing the risk of infection. Similarly, every client seen is given information on modes of HIV transmission and prevention. These clients are given demonstrations on condom use before, during and after sexual intercourse. Most clients are given monthly appointments and encouraged to come back whenever they require counseling or more condoms.

This study was a retrospective review of medical records of clients attended to at the Centre over a five-year period from January 2006 to December 2010.

The data extracted from the HCT Centre’s medical records included clients’ socio-demographic information, sexual behaviour, condom use and HIV testing results. Only the records with evidence of previous sexual exposure were included. Centre records with incomplete information and those outside the reference period were excluded. Effective condom use was defined as correct and consistent use of condom before during and after sexual intercourse. Consistent use is defined as using a condom for all acts of penetrative vaginal intercourse. Ineffective/non-use of a condom included slippage during intercourse or withdrawal, application of condom after genital contact, breakage and removal of condom before ejaculation or not using a condom at any stage during penetrative vaginal intercourse [10]. The collected data were entered, confirmed and analysed using SPSS version 15.0. Frequencies and proportions were used to summarise categorical variables, while quantitative data were presented as means and standard deviations. Bivariate analysis, using chi square statistics and crude odds ratio (COR) and their 95% confidence intervals (CIs) was used to identify factors associated with the main outcome variable non-use of condoms during the most recent act ofsexual intercourse. A multivariate logistic regression analysis was used to build a model of the outcome variable and the explanatory variables having p-values <0.2 on bivariate analysis. Adjusted odds ratios (AOR) and 95% CI were presented and used as measures of the strength of association.

Ethical approval to conduct the study was granted by the Ethics and Research Committee of the State Hospital, Osogbo. Confidentiality of client records was also assured.

## Results

One thousand nine hundred and twenty-one client records out of 2,108 were reviewed. One hundred and eighty seven records were excluded for lack of record of clients’ sexual exposure and lack of completeness. The mean age of the study population was 35.4 (SD 10.5) years (range 19–66 years). There were 1023 (53%) females and 898 (47%) males. Six hundred and forty eight (33.7%) had completed secondary education, the majority (62%) resided in urban areas and 232 (12%) were HIV positive (Table 1).

**Table 1:** Demographic characteristics of respondents

**Variable**	**Frequency of condom use (N=1921)**	**%**
**Age group (years)**		
18-24	229	12
25-34	751	39
35 and above	941	49
**Sex**		
Male	898	47
Female	1023	53
**Level of education**		
None	298	15
Primary	188	10
Secondary	722	38
Tertiary	717	37
**Marital status**		
Single	952	50
Married polygamous	535	28
Married monogamous	390	20
Widowed	44	2
**Place of residence**		
**Urban**	1191	62
**Rural**	730	38
**HIV status**		
**Positive**	232	12
**Negative**	1689	88

Only heterosexual vaginal sex was documented among the clients. Having multiple sexual partners was reported among 38.2% of the clients. Overall 45.2% of the clients did not use a condom in their last sexual act.

The relationship between selected attributes of clients and non-use of condom is shown in Table 2. About 44% of the clients with one sexual partner and 47% of those with multiple sexual partners did not use a condom during sex in their last sexual act (p=0.31). Also 45.4% of unmarried clients compared with 45% married clients did not use a condom during their last act of sexual intercourse (p=0.88).

**Table 2:** Bivariate analysis of selected variables and non-use of condom during most recent sexual act among the study population

**Variables**	**Proportion not using condom at last sexual intercourse (%)**	**COR**	**95% CI**	**p value**
**Age group (years)**				
18-24	148/229 (64.6)	2.80	2.08 -3.80	<0.001
25-34	349/751 (46.5)	1.33	1.10 - 1.62	<0.001
≥35	371/941 (39.4)	1		
**Sex**				
Female	482/1023 (47.1)	1.18	0.99 – 1.42	0.069
Male	386/898 (43.0)	1		
**Marital status**				
Single/widowed	454/1001 (45.4)	1.01	0.85 – 1.21	0.88
Married	414/920 (45.0)	1		
**Level of education**				
Secondary/tertiary (higher) education	624/1204 (51.8)	2.09	1.72 -2.53	<0.001
None/primary (lower) education	244/717 (34.0)	1		
**Number of sexual partners**				
**≥2 sexual partners**	342/733 (46.7)	1.10	0.92-1.32	0.31
**1 sexual partner**	526/1188 (44.3)	1		
**HIV status**				
**Positive**	172/232 (74.1)	4.09	3.00-5.57	<0.001
**Negative**	696/1689 (41.2)	1		

In the multivariate logistic regression model, the significant factors associated with non-use of condom at last sexual act were age group 18–24 years (AOR = 2.50, 95% CI = 1.83 – 3.42), age group 25 – 34 years (AOR 1.33, 95%CI 1.10 - 1.62), having attained higher education (AOR= 1.86, 95% CI = 1.52 – 2.26) and a positive HIV test result (AOR = 3.30, 95% CI = 2.40 – 4.55) (Table 3).

**Table 3:** Multivariate analysis of factors associated with non-use of condom during the most recent sexual act among respondents

**Variables**	**AOR; 95% CI; p value**
**Age group (years)**	
18 – 24	2.50; 1.83-3.42; <0.001
25 – 34	1.26 ; 1.03 – 1.54 <0.001
≥ 35	1
**Sex**	
Female	1.01 0.83 – 1.22 0.943
Male	1
**Education**	
Secondary/tertiary	1.86 1.52 – 2.26 <0.001
None/primary	1
**Number of sexual partner**	
≥ 2 partners	1.14 0.94 – 1.38 0.193
1 partner	1
**HIV results**	
Positive	3.30; 2.40 - 4.55; <0.001
Negative	1

## Discussion and conclusion

The study reviewed the clients’ records from the HCT Centre. It revealed that the majority of the clients attended to during the review period were young and sexually active. These are the characteristics of a population at risk of HIV and other sexually transmitted infections [7-9]. Therefore, it can be said that Osogbo HCT Centre is attending to the appropriate target population with a view to determining their HIV status and referring the HIV positive clients for treatment and follow-up while keeping the HIV negative clients negative thereby reducing HIV prevalence [7-9]. This study also showed that more female than male clients were attended to during the review period. This could be that female population was more receptive to information on HCT. Similarly, the females has been shown to be more affected by the HIV epidemic, as shown by various sentinel surveys worldwide [10-12]. For example, females constitute almost three-fifths (58.3% ) of the infected people in Nigeria [4,6]. Heterosexual vaginal sex with non-use of condom was reported, especially among the younger clients, and this could be responsible for the higher prevalence of HIV in this population. This practice, if left unchecked, will drive the spread of HIV further [13,14]. The effectiveness of latex condoms when properly used in preventing HIV/AIDS as well as other sexually transmitted infections (STIs) is well documented [15-17].

A higher proportion of married couples were recorded to have used a condom during their most recent act of sexual intercourse when compared to their unmarried counterparts, but this association was not statistically significant. This finding however raises the question of whether the partner at their most recent act of sexual intercourse was their spouse or somebody else. It also raises other questions on the reasons for condom use among married couples. Williamson et al., in a qualitative study of condom use among married couples in Kampala, Uganda in 2006, reported condom availability and a favourable environment as necessary for increasing condom use in their study population [18]. Also a high proportion of HIV transmission takes place between steady partners having unprotected sexual intercourse. Therefore, not using condoms or using them inconsistently can be a problem. This is particularly true in settings with high HIV prevalence, where the likelihood that a partner may be infected is higher . Previous studies have reported barriers to using condoms with steady partners or in stable relationships. These include trust and power inequalities. Also, the desire for children is a common issue among married couples, which can discourage condom use [19,20].

This study reported very high HIV prevalence among the study population. A previous study among these clients reported similar findings [21]. Furthermore, the non-use of condoms among the clients especially in clients with multiple partners implied low risk perception and could account for the high HIV prevalence among those clients. This study equally reported that being HIV positive was related to non-use of condom during the most recent act of sexual intercourse. This is an expected finding as HIV has been shown, in several studies, to be primarily transmitted in unprotected sexual intercourse with an infected partner and that effective use of condoms results in reduction in HIV transmission [10,22-24].

A higher level of education among the clients was also found to be related to non-use of condoms during the most recent act of sexual intercourse. This finding is surprising as clients with higher education were expected to have higher risk perception than the less educated clients. Further research is required in this area.

Findings in this study signify that the current effort to target at risk populations should be reinforced to combat spread of the HIV epidemic. Behavioral change communication interventions such as abstinence, faithfulness to one’s HIV negative partner, ensuring correct and consistent condom use during all acts of sexual intercourse, should be encouraged.

While interpreting the result presented in this study it may be important to consider factors that might have influenced our findings. This review of records relied on the Centre’s records some of which had to be excluded. The records relied on clients self-reporting their behaviour, which is a sensitive topic. Some clients may therefore have given socially acceptable response which differed from their actual behaviour. It could not be determined whether some clients or their partners were using other forms of contraception as this could have affected their condom use and sexual practices.

In conclusion, non-use of condoms during heterosexual intercourse was common among the study population, indicating a need to step up HIV preventive programme through a behavioural change communication strategy.

## Competing interest

The authors declare that they have no competing interests.

## Authors’ contributions

SAO and NAA made substantial contributions to conception and design of the study while all the authors were involved in data analysis and interpretation. All the authors were involved in writing the manuscript and approved the final copy.
